# Phytochemical, Antimicrobial, and Toxicological Evaluation of Traditional Herbs Used to Treat Sore Throat

**DOI:** 10.1155/2016/8503426

**Published:** 2016-06-26

**Authors:** Arifa Mehreen, Muzzamil Waheed, Iram Liaqat, Najma Arshad

**Affiliations:** ^1^Department of Zoology, University of the Punjab, Lahore, Pakistan; ^2^Faculty of Pharmaceutical Sciences, Government College University, Faisalabad, Pakistan; ^3^Government College University, Lahore, Pakistan

## Abstract

The* in vitro* antibacterial activities of 29 traditional medicinal plants used in respiratory ailments were assessed on multidrug resistant Gram-positive and Gram-negative bacteria isolated from the sore throat patients and two reference strains. The methanolic, n-hexane, and aqueous extracts were screened by the agar well diffusion assay. Bioactive fractions of effective extracts were identified on TLC coupled with bioautography, while their toxicity was determined using haemolytic assay against human erythrocytes. Qualitative and quantitative phytochemical analysis of effective extracts was also performed. Methanolic extract of 18 plants showed antimicrobial activity against test strains.* Adhatoda vasica* (ZI = 17–21 mm, MIC: 7.12–62.5 *μ*g/mL),* Althaea officinalis* (ZI = 16–20 mm, MIC: 15.62–31.25 *μ*g/mL),* Cordia latifolia* (ZI = 16–20 mm, MIC: 12.62–62.5 *μ*g/mL),* Origanum vulgare* (ZI = 20–22 mm, MIC: 3–15.62 *μ*g/mL),* Thymus vulgaris* (ZI = 21–25 mm, MIC: 7.81–31.25 *μ*g/mL), and* Ziziphus jujuba* (ZI = 14–20 mm, MIC: 7.81–31.25 *μ*g/mL) showed significant antibacterial activity. Alkaloid fractions of* Adhatoda vasica*,* Cordia latifolia*, and* Origanum vulgare* and flavonoid fraction of the* Althaea officinalis*,* Origanum vulgare*,* Thymus Vulgaris*, and* Ziziphus jujuba* exhibited antimicrobial activity. Effective plant extracts show 0.93–0.7% erythrocyte haemolysis. The results obtained from this study provide a scientific rationale for the traditional use of these herbs and laid the basis for future studies to explore novel antimicrobial compounds.

## 1. Introduction

Infectious diseases are a major cause of death and disability in humans as they are responsible for about 22% of the disease burden globally [1]. Sore throat is the most prevalent illness known to mankind. It has been reported that almost 25% of population experienced 2-3 episodes of infection every year [2].* Staphylococcus aureus* (*S. aureus*) is an opportunistic pathogen carried asymptomatically on the human body, mainly the anterior nares and throat [3]. Carriage of* S. aureus* plays a key role in the epidemiology and pathogenesis of infection and is associated with an increased risk of infectious complications after surgery in patients, intravascular devices, and superinfections [4]. Approximately 80% of invasive nosocomial infections are caused by strains of endogenous origin of nasal and throat [5, 6]. Antibiotics have saved lives of millions of people and contributed to improving quality and expectancy of life over the last century [7]. Since the discovery of penicillin in 1940s, antibiotics have been the best choice for the treatment of infectious diseases. However, the clinical efficacy of many presently used antibiotics is being threatened by the emergence of multidrug resistant (MDR) pathogens, as well as the use and misuse of existing antibiotics in humans, animals, and agriculture [8]. Several other factors like poverty, overcrowding, and lack of education all make this wonderful weapon useless. A number of multidrug resistant bacteria are increasingly observed in the normal community and hospital setting [9]. Methicillin-resistant* S. aureus* (MRSA) strains have acquired a gene that makes them resistant to all beta-lactam antibiotics. It is estimated that more people have died of MRSA infection than of other life threating diseases like HIV/AIDS and tuberculosis [10]. Hence, search for novel antimicrobial compounds or alternative therapy for these resistant infectious agents is inevitable.

Traditional herbal medicines have received much attention as a source of novel antibacterial drugs since they are considered as safe for human use [11]. Plant based medicines are widely used for primary health care in many developing countries [12]. As a result, it is found that about 60–80% of the world population relies on traditional treatment [13]. Plants have also been explored to get crude natural extracts for testing and developing potent and new antimicrobial drugs. A large number of secondary metabolites such as alkaloids, tannins, and flavonoids extracted from different medicinal plants have shown antimicrobial potential [14]. This finding has raised hope of obtaining novel antibiotics that can aid in fighting against multiple drug resistant bacteria [15].

For tracking and characterization of the active components thin layer chromatography (TLC) coupled with direct bioautography has gained the popularity as an effective technique [16]. Although TLC has a lower separation power than HPLC and GC, it offers several benefits such as limited samples preparation and ability to run many samples in parallel [17]. It has been proven to be effective, time-saving, and economical tool for bioassay-guided isolation of antibacterial components [18].

For the use of these herbs or their active part in human consumption, their safety towards human must be evaluated. Plants may contain such compounds that may have haemolytic or antihaemolytic effect on human erythrocytes. Therefore, many of the traditional plants need to be evaluated for their potential haemolytic activity to be categorised as a safer remedy to cure diseases.

The aims of the present study were (i) to screen the selected traditional herbs, chosen for the fact that they have been used in treating respiratory ailments or their symptoms, for potential antibacterial activity, (ii) to isolate active fraction(s), showing antibacterial activity by TLC direct bioautography, (iii) to carry out qualitative and quantitative phytochemical studies on active fractions, and (iv) to do toxicity analysis by determining the haemolysis percentage of the extract against human blood cells.

## 2. Experimental

### 2.1. Preparation of Plant Extract and Antimicrobial Efficacy

The fresh plant materials of selected plant (Table 1) were dried in open air protected from direct exposure to sunlight. Dried plant materials were separately powdered and extracted with 95% methanol or n-hexane using Soxhlet method, while aqueous extracts were prepared by soaking plant material in deionized water for 02-03 hours at 70°C. The extract so obtained was concentrated on rotary evaporator. The resulting material was dried to maximum possible level in freeze dryer and stored in glass vials at 4°C until used. For antimicrobial testing, 100 mg of the dry residue was dissolved in respective solvents or DMSO and evaluated through well diffusion assay against the six clinical and standard strains. Zone of inhibition was measured in mm and the breakpoint for susceptibility was taken as zone of inhibition >11 mm. Vancomycin and gentamicin were used as positive control, while DMSO was employed as a negative control.

### 2.2. Bacterial Strains

Methicillin-resistant and methicillin-susceptible* S. aureus* and* Pseudomonas aeruginosa* (*P. aeruginosa*) strains were isolated from sore throat patients from tertiary care hospitals at Faisalabad. ATCC strains of* Escherichia coli* (*E. coli*) and* S. aureus* were obtained from lab stock. All strains were routinely grown and identified. For further use they were preserved at −20°C.

### 2.3. Antimicrobial Susceptibility of Clinical Isolates

Antibiotic sensitivity of the isolated* S. aureus* strains was determined by Standard Disc Diffusion Method [19]. Different antibiotics (Oxoid) were used in the present work: tetracycline (30 *μ*g), vancomycin (30 *μ*g), clindamycin (2 *μ*g), methicillin (5 *μ*g), cefixime (5 *μ*g), erythromycin (15 *μ*g), oxacillin (1 *μ*g), gentamicin (10 *μ*g), streptomycin (10 *μ*g), chloramphenicol (30 *μ*g), linezolid (10 *μ*g), ampicillin-sulbactam (20 *μ*g), and penicillin (10 *μ*g) [20].

### 2.4. Minimum Inhibitory Concentration (MIC)

Minimum inhibitory concentrations (MIC) of antibiotics and plant extracts were determined by the microdilution method as described by Clinical and Laboratory Standards Institute (formerly the National Committee for Clinical Laboratory Standards, NCCLS) [20]. The antibiotic was serially diluted in Mueller-Hinton broth in 96-well plates. The plant extracts solutions were separately added to wells in a final concentration of 1 mg/mL; then bacterial inoculum size of 105 CFU/mL was added to each well. Controls without plant extracts, without bacterial inoculum, or with plant extracts only were also included in the experiment. Each plant extract was run in duplicate. The test plates were incubated at 37°C for 24 h. The MIC was taken as the minimum concentration of the dilutions that inhibited the growth of the test microorganism. The growth was recorded in terms of button formation in wells; it was confirmed by adding tetrazolium chloride.

### 2.5. Toxicity of Extracts to Human Erythrocytes

The cellular toxicity of the extracts from different plants was determined [21]. Erythrocytes were isolated from human blood by removing plasma and buffy coat and suspended in phosphate buffered saline (10 mM phosphate, 150 mM sodium chloride) making a final concentration of 2% erythrocytes. The dilutions of plant extract (100 mg/mL) were made and mixed with erythrocytes keeping the final volume up to 1 mL. The cells were incubated for 1 hr at 37°C and finally centrifuged at 1500 rpm for 10 minutes [22]. The lysis of the cells was observed by determining absorbance at 540 nm using spectrometer. Cell in distilled water was taken as negative and cells suspended in normal saline were taken as positive control. The mixture was centrifuged at 1500 rpm for 1 minute in a laboratory centrifuge. The free haemoglobin in the supernatant was measured at 540 nm.

The haemolysis percentage was calculated by the following formula:

(1) $$\begin{array}{c} \%\text{haemolysis}=\frac{At-An}{Ac-An}*100. \end{array}$$

At is absorbance of test sample, An is absorbance of the control (saline), and Ac is absorbance of the control (water).

### 2.6. Screening and Estimation of Some Phytochemical Components

Phytochemical screening of the effective extract for the detection of alkaloids, flavonoids, steroids, terpenoid, and other secondary metabolites was carried out by following the procedure of Trease and Evans [23]. Total alkaloids, flavonoids, and saponin fraction were also separated and their antimicrobial activity was carried out [24].

### 2.7. Thin Layer Chromatography, Bioautography, and Identification of the Chemical Nature of the Bioactive Compound

For TLC, 10–20 *μ*L of plant extract was loaded on silica gel sheet (Merck, Darmstadt, Germany). Different solvent systems, chloroform : methanol (80 : 20), n-butanol : acetic acid : water (4 : 1 : 1), and acetone : methanol (1 : 1), were used as mobile phase. The TLC plates (a–f) were run in triplicate. Plate “a” was used to determine the spots by visualizing in UV light to see if the separated spot was UV active after which it was sprayed with vanillin sulphuric acid reagent (2%) to detect all the separated spots. Plate “b” was used for autobiography. Agar overlay method [25] was used for direct bioautographic assay, with little modification, to detect antimicrobial fractions in plant extracts which were active against clinical sample of MRSA and* E. coli*. Soft nutrient agar (1%) was seeded with 10^6^ CFU/mL of MRSA/*E. coli* and overlaid on TLC plate. It was then incubated overnight in a controlled environment at 37°C. Subsequently, the plates were sprayed with 2,3,5-triphenyltetrazolium chloride and further incubated for three hours at 37°C. Microbial growth inhibition appeared as clear zone against a pink background. The Rf value of the bioactive spots was measured as the ratio of mobility of centre of a bioactive spot against the total distance travelled by the solvent front. The bioactive spots were scraped from the TLC plate “c” and eluted in 500 *μ*L ethanol. The solution was filtered using Whatman filter paper number 1 and concentrated and again bioassay was performed to recheck the activity. Plates “d, e, and f” were sprayed separately with TLC reagents including FeCl3 (10%), Dragendorff's reagent, and KOH (5N) to detect the presence of phenolic compounds, alkaloids, and flavonoids, respectively, in bioactive spots.

## 3. Results

### 3.1. Antibiotic Susceptibility and Responses to Plant Extracts

All clinical isolates and ATCC* E. coli* were resistant to beta-lactam group, whereas ATCC 25923 was sensitive to all antibiotics used in the study. The clinical isolates were also resistant to diverse groups of antibiotics (Table 2). Aqueous and n-hexane extracts displayed antimicrobial activity with ZI < 11 mm, while methanolic extracts of 18/29 plants were found to be active and showed varying activity with a zone of inhibition of 11–25 mm for all the clinical and reference strains. The MIC of the extracts ranged from 3.90 to 250 *μ*g/mL (Table 3).

### 3.2. Phytochemical Analysis

The plant extracts which showed promising antimicrobial activity were investigated further for the presence of flavonoids, terpenoids, steroids, and glycosides, and other phytochemicals results are given in Table 4. Alkaloids, flavonoids, and saponin fraction were separated. MIC and their bioactivity were checked out (Table 5). Alkaloids fraction of* Adhatoda vasica*,* Cordia latifolia*, and* Origanum vulgare* and flavonoid fraction of* Althaea officinalis*,* Origanum vulgare*,* Thymus vulgaris*, and* Ziziphus jujuba* displayed antimicrobial activity against MRSA. MIC of the alkaloids and flavonoids ranged from 3.25 to 12.5 (*μ*g/mL) and zone of inhibition ranged from 13 to 18 mm.

### 3.3. Thin Layer Chromatography and Autobiography

Different solvent systems comprising water, methanol, acetic acid, chloroform, n-butanol, toluene, ethyl acetate, and formic acid in different combination were used to separate the active part. The best solvent systems were chloroform and methanol (80 : 20), n-butanol, acetic acid, and water (4 : 1 : 1). Active parts of all the plant extract were not separated in a single solvent system which gives us the information that the active fractions vary in their chemical nature. Antimicrobial fractions of the crude extract were separated by TLC followed by autobiography method. The Rf value of active fraction is shown in Table 6. When TLC plate was visualized under UV different coloured spots were seen and marked and their antimicrobial activity was checked out. The chemical nature of the antimicrobial compound was detected by spraying with Dragendorff's reagent for alkaloids and 10% FeCl3 for phenolic compound and 5N KOH solution for flavonoids.

Thin layer chromatography plates after the development show various components in light and when visualized under UV other parts were also visualized. Direct autobiography on TLC plates revealed presence of active antimicrobial components in all six plants with different Rf values (Table 6).

### 3.4. Haemolysis Percentage of the Crude Methanolic Extract

*In vitro* evaluation of the toxicity of the extract by comparing the haemolysis percentages is shown in Figure 1. It has been shown in the graph that the maximum haemolytic activity was shown by methanolic extract of the* Cordia latifolia* and the minimum haemolytic activity was shown by* Origanum vulgare*. On the basis of haemolytic potential the selected plants could be arranged as follows:* Cordia latifolia* >* Ziziphus jujuba* >* Althaea officinalis * = * Adhatoda vasica* >* Thymus vulgaris* >* Origanum vulgare*.

## 4. Discussion

The interest in research on medicinal plants has increased over the last few decades due to the emergence of MDR strains of important pathogens like* S. aureus*,* P. aeruginosa*, and* E. coli* [26]. Some of the antibiotics against which resistance has been developed include penicillin G, macrolides, lincosamides, tetracycline, and gentamicin [27]. Investigations are needed for antibacterial agents that offer broad-spectrum activity against resistant strains of microorganisms. Toxicity profiling of the plant extract also needs scientific validation.

In the present study, twenty-nine plants that were recommended by herbal practitioners for treatment of diseases related to respiratory tract were evaluated for their antibacterial activity against MDR strains of* S. aureus*,* E. coli*, and* P. aeruginosa* isolated from sore throat patients. Although the antibacterial effect of these plants has already been reported by many workers, their activities against MDR strains are less evaluated [28–31]. Moreover, the current study focused on the phytochemical nature of active fraction. Three types of extracts, n-hexane, water, and methanol, were tested for their possible antibacterial activity against ATCC bacterial cultures of Gram-positive and Gram-negative bacteria and clinical samples of MDR* S. aureus* and* P. aeruginosa* isolated from the sore throat patients. A zone of inhibition of >11 mm was considered as a standard for effectiveness of extract against bacteria. The n-hexane extracts did not show any zone of inhibition, while aqueous extract inhibits microbial growth with a zone of inhibition of less than 11 mm. Although the aqueous extract preparation mimics the traditional method of use, very little antimicrobial activity was observed in it, which might be due to less solubility of active components in water [32, 33]. On the other hand methanolic extract of 18/29 plants exhibits ZI > 11 mm and MIC of 3.91–500 *μ*g/mL, indicating that methanolic extract contains a variety and better quantity of bioactive compounds. Such observation has also been noticed by some workers [34, 35].

Plants extracts having MIC ≤ 100 *μ*g/mL against all test strains were selected for detailed study including phytochemical analysis (qualitative and quantitative), TLC, autobiography, and* in vitro* toxicity. Qualitative analysis revealed the presence of alkaloids, flavonoids, terpenoids, steroids, saponin, tannins, carbohydrates, proteins, cardiac glycosides, phenols, and reducing sugars. The saponin, alkaloids, and flavonoids are documented as the most active ingredients to which the antimicrobial activities of many plant species can be attributed [36]. Therefore, quantitative analysis was carried out for these. Moreover, their rich fractions were verified to be responsible for antibacterial activity against test strains.

*Adhatoda vasica* contained bioactive alkaloid (2%) fraction. On TLC plates, three spots were noticed by bioautography which separated at 0.4, 0.86, and 0.92 Rf values in chloroform : methanol (80 : 20) solvent system. One of the spots was identified as alkaloid, while chemical nature of other 2 spots could not be determined.* Adhatoda vasica* has also been recognized for its diverse health benefits along with antimicrobial potential. Kaur et al. [37] and Sawant et al. [38] have recently reported antimicrobial activity against respiratory pathogens* S. aureus* and* E*.* coli*. The differences may be due to strain specificity or geographical variations in plant spp. Alkaloids l-vasicinone, deoxyvasicine, maiontone, vasicinolone, and vasicinol were reported in* Adhatoda vasica* by Jain and Sharma [39]. The current study indicates that it is not only alkaloid that shows antimicrobial activity; some other compounds of different nature are also bioactive and further studies are required for their separation and identification.

*Origanum vulgare* contained bioactive alkaloid (1.5%) and flavonoid (2.5%) fraction. On TLC plates, three spots were noticed by following autobiography which separated at Rf 0.75, 0.79, and 0.82 values in butanol : acetic acid : water (4 : 1 : 1) solvent system. One of the spots with Rf value of 0.79 was identified as alkaloid and another one with Rf value of 0.82 was identified as flavonoid, while chemical nature of the third spot could not be determined.* Origanum vulgare* and its EO have also been recognized for its antimicrobial and antioxidant nature [40]. The current study indicates that alkaloid and flavonoids as well as other compounds with antimicrobial potential can be purified from* Origanum vulgare* and used against MDR.

*Thymus vulgaris* leaves and essential oil are used in cosmetic and food additives [41, 42]. Antimicrobial potential of thymus was also reported [43, 44], but nature of component was not known. In this study, phenolic compound with Rf value of 0.72 was found responsible for antibiotic activity, while another of unknown nature was also bioactive.

Flavonoid of* Ziziphus* displayed antimicrobial activity. Recently published data on antimicrobial properties against Gram-positive and Gram-negative pathogenic bacteria have been reported [45], whereas the presence of alkaloids, flavonoids, and saponin in* Ziziphus jujuba* extracts was reported by [46]. The current study confirms antimicrobial nature of its flavonoid. TLC plate separation leads to identification of 5 spots with bioautography of Rf value of 0.15, 0.18, 0.65, 0.71, and 0.85 through autobiography. Among them 3 were phenolic; one of them was flavonoid, whereas chemical nature of one spot with Rf of 0.85 remained unclear. The current study indicates that the flavonoids with Rf of 0.45 and one compound with Rf of 0.72 have this activity. In a review presence of a variety of flavonoids in the methanolic extract was reported by Gao et al. [47].

TLC separation of methanolic extract of* Cordia latifolia* showed 03 bioactive spots with Rf value of 0.84, 0.67, and 0.35. The alkaloid fraction of the methanolic extract with Rf value of 0.84 and other two spots with Rf value of 0.67 and 0.35 of unknown nature show antibacterial activity.

Scientific validations of the safety of extracts are mandatory for recommendation to human. The erythrocyte haemolysis has been widely used as an indicator of toxicity of injectable formulations as well as a general indication of membrane toxicity. Haemolysis is due to red blood cells destruction which resulted from lysis of membrane lipid bilayer. This haemolysis relates to concentration and chemical composition of extract. Data about the safety of* Cordia latifolia* and* Althaea officinalis* has been provided by May and Willuhn [48] and Caparroz-Assef et al. [49]. Extracts of* Adhatoda vasica*,* Althaea officinalis*,* Oregano vulgaris*,* Cordia latifolia*,* Althaea officinalis*, and* Thymus vulgaris* were used in toxicity study and revealed 0.93–6.48% haemolytic activity and are found to be safe for human use.

## 5. Conclusion

In conclusion 29 plants included in the study were already known for their antimicrobial nature; the current study found that 18/29 possess these characteristics against MDR strains and 6/18 are good candidates for isolation of effective components.* Cordia latifolia*,* Ziziphus jujuba*,* Althaea officinalis*,* Adhatoda vasica*,* Thymus vulgaris*, and* Origanum vulgare* have good antimicrobial activity and their haemolysis assay declared them safe candidate for the treatment of sore throat in human. Alkaloids of* Adhatoda vasica*,* Cordia latifolia*, and* Origanum vulgare* and flavonoids of* Althaea officinalis*,* Origanum vulgare*,* Thymus vulgaris*, and* Ziziphus jujuba* may be utilized for the treatment of MRSA.

## Figures and Tables

**Figure 1:** Toxicity of methanolic extracts of selected plants against human erythrocytes.

**Table 1:** List of plants used in herbal medicine for the treatment of sore throat.

Serial number	Plant name	Family name	Common name	Part of plant used	Voucher number
1	*Adhatoda vasica *(L.)	Acanthaceae	Nees	Leaves	ZD-IM-01
2	*Aloe vera *(L.)	Xanthorrhoeaceae	Alovera	Leaves	ZD-IM-02
3	*Althaea officinalis *(L.)	Malvaceae	Marshmallow	Flowers, leaves	ZD-IM-03
4	*Cinnamomum zeylanicum *(L.)	Lauraceae	Cinnamon	Bark	ZD-IM-04
5	*Cordia latifolia *(Roxb.)	Boraginaceae	Sapistan, lasori	Fruits	ZD-IM-05
6	*Emblica officinalis *(Gaertn.)	Euphorbiaceae	Indian gooseberry	Fruits	ZD-IM-06
7	*Eugenia caryophyllata *(L.)	Myrtaceae	Clove	Fruit	ZD-IM-07
8	*Glycyrrhiza glabra *(L.)	Leguminosae	Liquorice	Roots	ZD-IM-08
9	*Hyssopus officinalis *(L.)	Lamiaceae	Hyssop	Leaves, flowers	ZD-IM-09
10	*Lawsonia inermis *(L.)	Lythraceae	Henna	Leaves	ZD-IM-10
11	*Linum usitatissimum *(L.)	Linaceae	Flax seed	Seed	ZD-IM-11
12	*Malva sylvestris *(L.)	Malvaceae	Mallow	Flowers	ZD-IM-12
13	*Matricaria chamomilla *(L.)	Asteraceae	Chamomile	Flowers	ZD-IM-13
14	*Mentha piperita *(L.)	Lamiaceae	Mint	Leaves	ZD-IM-14
15	*Moringa oleifera *(Lam.)	Moringaceae	Moringa, drumstick tree	Leaves	ZD-IM-15
16	*Morus alba *(L.)	Moraceae	White mulberry	Fruits, leaves	ZD-IM-16
17	*Ocimum basilicum *(L.)	Labiatae	Basil	Leaves	ZD-IM-17
18	*Onosma bracteatum *(L.)	Boraginaceae	Gao zuban	Leaves, flowers	ZD-IM-18
19	*Origanum vulgare *(L.)	Labiatae	Oregano	Leaves	ZD-IM-19
20	*Pimpinella anisum *(L.)	Umbelliferae	Anise	Fruit	ZD-IM-20
21	*Piper longum *(L.)	Piperaceae	Long pepper	Fruit	ZD-IM-21
22	*Saussurea lappa *(L.)	Compositae	Kuth	Root	ZD-IM-22
23	*Sisymbrium irio *(L.)	Brassicaceae	London rocket	Seeds	ZD-IM-23
24	*Syzygium cumini *(L.)	Myrtaceae	Jambolan	Fruit, leaves	ZD-IM-24
25	*Thymus vulgaris *(L.)	Lamiaceae	Thyme	Leaves	ZD-IM-25
26	*Viola odorata *(L.)	Violaceae	Sweet violet	Leaves, flowers	ZD-IM-26
27	*Vitis vinifera *(L.)	Vitaceae	Grapes	Leaves, fruits	ZD-IM-27
28	*Zingiber officinale *(Roscoe)	Zingiberaceae	Ginger	Root	ZD-IM-28
29	*Ziziphus jujuba *(mill.)	Rhamnaceae	Red date	Fruit	ZD-IM-29

The plants materials were dried in shades, identified by the help of Dr. Muhammad Nasir (Taxonomist, Department of Botany, University of the Punjab), and kept in Microbiology and Immunology Laboratory (Department of Zoology, University of the Punjab) under the voucher numbers listed above.

**Table 2:** Antibiogram of the clinical and standard bacteria.

Clinical sample	Resistant	Intermediate	Sensitive
S1	Me, cef, eryth, oxa, strep, amp, pen	No	Tet, vanco, clind, genta, chlo, lin
S2	Tet, clin, me, cef, ery, oxa, chlo, amp, pen	None	Van, gen, strep, lin
S3	Tet, me, cef, oxa, gen, pen	None	Van, clin, ery, strep, chlo, lin, amp
*P. aeruginosa *	me, cef, oxa, gen, pen, ery	Tet, clin, amp	Van, clin, strep, chlo, lin
*E. coli *ATCC 8739	Me, pen	None	Tet, cef, oxa, gen, Van, clin, ery, strep, chlo, lin, amp
*S. aureus *ATCC 25923	None	None	Tet, me, cef, oxa, gen, pen, Van, clin, ery, strep, chlo, lin, amp

**Table 3:** MIC/MBC of plant extracts against selected bacteria.

Serial number	Plant name	S1		S2		S3		*P. aeruginosa*		*S. aureus* (25293)		*E. coli* (8739)	
		ZI	MIC *µ*g/mL	ZI	MIC	ZI	MIC	ZI	MIC	ZI	MIC	ZI	MIC
*1*	*Adhatoda vasica*	17	31.25	18	31.25	21	31.25	19	62.5	21	7.81	18	31.25
*2*	*Althaea officinalis*	16	31.25	18	31.25	20	31.25	20	31.25	20	15.63	20	31.25
*3*	*Cinnamomum zeylanicum*	20	250	22	125	25	7.81	20	125	25	125	22	250
*4*	*Cordia latifolia*	16	31.25	18	62.5	20	31.25	17	125	20	12.63	19	62.50
*5*	*Emblica officinalis*	11	125	12	250	13	125	13	125	13	62.50	12	250
*6*	*Glycyrrhiza glabra*	18	125	20	250	22	125	17	62.50	22	31.25	19	125
*7*	*Hyssopus officinalis*	18	125	19	250	22	125	18	31.25	22	31.25	18	62.50
*8*	*Lawsonia inermis*	12	250	13	250	15	250	14	125	15	125	13	250
*9*	*Linum usitatissimum*	21	250	22	250	22	250	19	125	22	125	20	250
*10*	*Malva sylvestris*	15	125	16	250	18	125	15	62.5	18	62.50	16	125
*11*	*Matricaria chamomilla*	12	125	13	250	14	125	13	62.5	13	62.50	15	125
*12*	*Moringa oleifera*	13	250	14	500	15	250	15	62.5	15	62.50	14	250
*13*	*Morus alba*	13	125	12	250	13	125	13	125	13	31.25	13	125
*14*	*Origanum vulgare*	22	7.81	20	15.62	22	7.81	20	7.81	22	3.91	21	15.63
*15*	*Sisymbrium irio*	20	125	22	250	25	125	21	62.5	25	62.50	20	125
*16*	*Syzygium cumini*	13	62.5	13	125	15	62.50	13	31.25	15	15.63	13	62.50
*17*	*Thymus vulgaris*	22	15.63	22	31.25	25	15.63	22	7.81	25	7.81	21	31.25
*18*	*Ziziphus jujuba*	14	15.63	14	31.25	12	15.63	21	7.81	14	7.81	16	31.25

**Table 4:** Phytochemical analysis of the methanolic extracts of plants possessing antibacterial activity.

Serial number	Plant name	Yield %	Alk.	Flv.	Ter.	Ste.	Sap.	Tan.	Carb.	Pro.	Car. Gly.	Phe.	Red. Sug.
1	*Adhatoda vasica*	18.2	+	+	+	−^*∗∗*^	+	+	−	+	+	+	+
2	*Althaea officinalis*	22	−	+	−	++^*∗*^	−	++	++	+	++	++	++
3	*Cordia latifolia*	29.9	+	−	−	−	−	++	++	++	−	−	−
4	*Origanum vulgare*	35.6	+	+	−	+	+	−	−	+	+	+	+
5	*Thymus vulgaris*	22.9	−	+	−	−	−	−	−	+	−	+	−
6	*Ziziphus jujuba*	22.5	−	+	+	+	−	−	+	−	−	+	+

Tan., tannins; Alk., alkaloids; Flv., flavonoids; Ter., terpenoids; Ste., steroids; Sap., saponins; Carb., carbohydrate; Pro., proteins; Car. Gly., cardiac glycosides; Phe., phenols; Red. Sug., reducing sugar.

++^*∗*^: high concentration.

−^*∗∗*^: absence.

**Table 5:** Bioactivity of secondary metabolites rich fraction.

Serial number	Plant name	Alkaloid			Flavonoid			Saponin		
		ZI (mm)	MIC (*µ*g/mL)	% age estimation	ZI (mm)	MIC (*µ*g/mL)	% age estimation	ZI (mm)	MIC (*µ*g/mL)	% age estimation
1	*Adhatoda vasica*	13	6.25	2	0	>100	—	0	>100	—
2	*Althaea officinalis*	—	N.D^*∗*^	N.D	14	12.5	1.03	0	>100	2.7
3	*Cordia latifolia*	14	12.5	0.8	0	N.D	—	0	N.D	—
4	*Origanum vulgare*	18	6.25	1.5	15	3.25	2.5	—	N.D	—
5	*Thymus vulgaris*	—	N.D	—	16	6.25	2.3	—	N.D	—
6	*Ziziphus jujuba*	—	N.D	—	13	6.25	1.33	—	N.D	—

^*∗*^N.D: activity not determined.

**Table 6:** Retention factor of the antibacterial fraction of the methanolic crude extract.

Serial number	Plant name	Rf^*∗*^ value Cm	Mobile phase
1	*Adhatoda vasica*	0.4 (alkaloids) 0.86 0.92	Chloroform : methanol (80 : 20)

2	*Ziziphus jujuba*	0.15 (phenol) 0.18 (flavonoids) 0.65 (phenol) 0.71 (phenol) 0.85	Chloroform : methanol (80 : 20)

3	*Althaea officinalis*	0.72 0.45 (flavonoids)	Chloroform : methanol (80 : 20)

4	*Cordia latifolia*	0.67 0.84 (alkaloids) 0.35	Acetone : methanol (1 : 1)

5	*Origanum vulgare*	0.75 0.79 (flavonoids) 0.82 (alkaloids)	Butanol : acetic acid : water (4 : 1 : 1)

6	*Thymus vulgaris*	0.72 (phenol) 0.8	Butanol : acetic acid : water (4 : 1 : 1)

^*∗*^Retention factor.
